The article "Identification of Key Genes in Severe Burns by Using Weighted Gene Coexpression Network Analysis" was published in 2022. Journal: Comput Math Methods Med.

# Identification of Key Genes in Severe Burns by Using Weighted Gene Coexpression Network Analysis

**DOI:** 10.1155/2022/5220403

**Published:** 2022-06-28

**Authors:** ZhiHui Guo, YuJiao Zhang, ZhiGuo Ming, ZhenMing Hao, Peng Duan

**Affiliations:** Burns Department, General Hospital of TISCO, Taiyuan, 030003 Shanxi, China

## Abstract

The aims of this work were to explore the use of weighted gene coexpression network analysis (WGCNA) for identifying the key genes in severe burns and to provide a reference for finding therapeutic targets for burn wounds. The GSE8056 dataset was selected from the gene expression database of the US National Center for Biotechnology Information for analysis, and a WGCNA network was constructed to screen differentially expressed genes (DEGs). Gene Ontology and pathway enrichment of DGEs were analyzed, and protein interaction network was constructed. A burn mouse model was constructed, and the burn tissue was taken to identify the expression levels of differentially expressed genes. The results showed that the optimal soft threshold for constructing the WGCNA network was 9. 10 coexpressed gene modules were identified, among which the green, brown, and gray modules had the largest number of burn-related genes. The DEGs were mainly related to immune cell activation, inflammatory response, and immune response, and they were enriched in PD-1/PD-L1, Toll-like receptor, p53, and nuclear factor-kappa B (NF-*κ*B) signaling pathways. 5 DEGs were screened and identified, namely, Jun protooncogene (JUN), signal transducer and activator of transcription 1 (STAT1), BCL2 apoptosis regulator (Bcl2), matrix metallopeptidase 9 (MMP9), and Toll-like receptor 2 (TLR2). Compared with skin tissue of normal mouse, the messenger ribose nucleic acid (mRNA) and protein expression levels (PEL) of STAT1 and Bcl2 in burn tissue were greatly decreased, while those of JUN, MMP9, and TLR2 were increased obviously (*p* < 0.05). In conclusion, STAT1, Bcl2, JUN, MMP9, and TLR2 can be potential biological targets for the treatment of severe burn wounds.

## 1. Introduction

Burn is a very special trauma, and its incidence is closely related to emergencies, traffic accidents, and daily life [1]. Severe burns can result in the loss of limb function and even death [2]. Burn patients will suffer physical and psychological harm if they receive a significant number of skin grafts, harsh physical therapy, or long-term rehabilitation treatment [3, 4]. Large-scale burns will cause a series of immunological and pathophysiological changes in the body, which will eventually lead to the disorder of the immune system [5]. Therefore, some scholars believe that the disturbance of immune system function after burn is an important factor leading to severe infection, multiorgan/system dysfunction, or death after burn [6]. Factors such as large-area tissue necrosis, stress response, shock, infection, or nutritional deficiency after burns, together with subsequent treatment, will change the microenvironment of immune cells in the body [7, 8]. Therefore, although burn treatment techniques can improve the clinical symptoms and prognosis of patients to a certain extent, they cannot reduce the mortality of patients [9]. Therefore, it is urgent to understand the specific mechanism of maintaining and regulating immune dysfunction in burn patients and to find corresponding treatment methods.

Because gene chip and sequencing technologies can directly examine transcriptome data, it has become the primary tool for investigating the molecular mechanisms underlying life activities [10]. It is difficult to dig out the underlying molecular mechanisms by simply analyzing the transcriptome of a single tissue or sample. However, analyzing biological networks can reflect the interaction between different biomolecules at the system level, but cannot provide possibilities for exploring complex biological phenomena [11]. Weighted gene coexpression network analysis (WGCNA) can identify coexpression modules in multiple biological samples based on the correlation between different gene expression profiles and find coexpression modules that are highly related to them after phenotypic correlation [12]. Compared with other coexpression analysis methods, the WGCNA network uses a soft threshold method to provide the sensitivity of the network to module identification, so the network has been widely used in the analysis of coexpression patterns in various organisms [13, 14]. The approach uses an approximate scale-free topology to generate the soft threshold and then replaces the previous traditional algorithm's hard threshold [15–18].

Therefore, the WGCNA method is adopted systematically to explore the expression patterns of severe burn tissue and normal tissue in this work, aiming to find the key genes of severe burn wound healing and provide a molecular-level theoretical basis for the search for clinical therapeutic targets of burn wounds.

This paper is organized as follows: Section 2 presents the materials and methods of the proposed concepts.  Section 3 describes the statistical analysis and results.  Section 4 presents the discussion of the whole paper.  Section 5 summarizes this paper and offers directions for future work.

## 2. Materials and Methods

### 2.1. Basis of the WGCNA Algorithm

WGCNA belongs to a class of gene coexpression networks. The algorithm introduces an approximate scale-free topology to accurately calculate the soft threshold and then replaces the hard threshold of the previous traditional algorithm [15]. Compared with random networks, scale-free topology is more realistic. After standardization of the experimental data, WGCNA analysis can be performed. The specific analysis process is shown in Figure 1.

The coexpression network was adopted to construct a matrix *A* of the expression levels of samples and related genes. It was assumed that the gene was represented by *i*, and the sample size detection value was *j*; the mathematical expression of the matrix could be given as follows:

(1) $$\begin{array}{c} A=\left\{a_{ij}\right\}=\left\{a_{1},a_{2},\cdots ,a_{n},\right\}. \end{array}$$

After transformation of expression profile data matrix and calculation of the correlation between genes using matrix operations, the coexpression similarity can be defined using the absoluteness of the correlation coefficient:

(2) $$\begin{array}{c} {\text{Similarity}}_{ij}=\left|\text{cor}\left(a_{i},a_{j}\right)\right|. \end{array}$$

In Equation (2) above, Similarity_*ij*_ represented the similarity of the expression profiles of genes *i* and *j*, and the value ranged from 0 to 1.

The similarity matrix was converted to an adjacency matrix, and then, the WGCNA weighting coefficient *β* could be determined based on the Pareto distribution law:

(3) $$\begin{array}{c} N_{ij}={\text{Similarity}}_{ij}^{\beta }. \end{array}$$

In the above Equation (3), *N*_*ij*_ was an adjacency matrix, and *β* was a weighting coefficient or a soft threshold.

To determine the dissimilarity of the highly connected gene forming modules in the constructed network, the adjacency matrix can be converted into a topological matrix, and then, topological reconstruction can be selected to calculate the degree of intergene association. The equation for calculating topological overlap was defined as follows:

(4) $$\begin{array}{c} \omega_{ij}=\frac{L_{ij}+N_{ij}}{\min\left\{k_{i},k_{j}\right\}+1-N_{ij}}, \end{array}$$

(5) $$\begin{array}{c} L_{ij}=\underset{u}{\sum }n_{iu}n_{ju}. \end{array}$$

In Equation (4) above, *L*_*ij*_ was the sum of the products of adjacency coefficients of gene *i* and *j* connecting nodes, and *k* referred to the sum of adjacency coefficients of gene connecting nodes. When *ω*_*ij*_ = 1, it meant that genes *i* and *j* were connected to all genes; when *ω*_*ij*_ = 0, it meant that genes *i* and *j* were not connected to all genes.

The WGCNA required to use the dissimilarity calculated by the topological overlap method for hierarchical clustering and then obtain different gene modules of different branches [16]. The dynamic pruning was applied for the construction of cluster numbers to mine more modules. Gene coexpression network was to use systems biology methods to search for highly correlated modules. WGCNA can continuously approximate genes into a scale-free topology network through a weighted method and then construct a coexpression network and find hub genes in modules of interest [17]. Hub genes can be searched by threshold setting or by using function network screening.

### 2.2. Selection of Materials for WGCNA

The microarray data related to burns were screened from the gene expression database of the National Center for Biotechnology Information (NCBI) (http://www.ncbi.nlm.nih.gov/geo/), and GSE8056 was finally selected as the research object according to the research subjects and sample size. The samples in this dataset were derived from the skin samples of burn patients quickly obtained in the operating room and then detected and analyzed by high-throughput chips. The dataset contained a total of 12 samples, which were the normal group (accession numbers: GSM198875, GSM198876, and GSM198877) and the burn group (accession numbers: GSM198866, GSM198867, GSM198868, GSM198869, GSM198870, GSM198871, GSM198872, GSM198873, and GSM198874). Relevant gene records with *p* values less than 0.05 were selected and included in the WGCNA.

### 2.3. Construction of WGCNA

The “Flash Clust” software in the R language package was used for cluster analysis of the included samples, and the “Pick Soft Threshold” function was to adjust the weight of the weighting coefficient *β*. The matrix with correlation and adjacent relationship was calculated as a topological overlap matrix (TOM) using WGCNA, and the dissimilarity was calculated. The dissimilarity was undertaken as a distance metric to perform hierarchical clustering of genes and obtain identification modules, cluster markers, and merge highly similar modules. The “Plot Dendro and Color” function was selected to visualize the gene module and select the target genes within the module to draw a heat map. Finally, the genes in the modules closely related to severe burn were found, and the cluster analysis of the relationship heat map was performed on the clinical characteristics. The specific flow of burn-related gene analysis using WGCNA is shown in Figure 2.

### 2.4. Screening of DEGs

Background correction of raw data was performed using robust multiarray average software, and DEGs were obtained using independent samples *t*-test and fold method. Comparative analysis of DEGs in burn tissue and normal tissue was performed using the analysis tool that came with the gene expression database in the NCBI dataset. The screening conditions were set as:

1. The corrected *p* value (the adj *p* value) was less than 0.05
2. The absolute value of the log gene expression fold difference (|logFC|) was ≥1.5

### 2.5. Analysis on Gene Ontology and Pathway Enrichment of DEGs

Gene Ontology can be used for functional annotation of genes. The functional enrichment analysis of Gene Ontology included molecular function (MF), biological process (BP), and cellular component (CC). The gene set enrichment analysis software and profiler online tool were adopted in this work for enrichment analysis and annotations of the module and Kyoto Encyclopedia of Genes and Genomes (KEGG).

### 2.6. Construction and Analysis on Protein Interaction Network of DEGs

The STRING database can be selected to predict the functional correlation between proteins, and its prediction accuracy for genes was as high as 80% or more. The protein-protein interaction network of DEGs obtained by screening was constructed using the STRING 11.0 online tool (https://cn.string-db.org/). Protein interactions with confidence greater than 0.5 were selected from the protein-protein interaction network. The DEGs protein interaction network was constructed using Cytoscape software.

### 2.7. Identification of DEGs

#### 2.7.1. Construction of Burn Animal Model

20 healthy adult BALB/c mice, male or female, were selected as research subjects. Mice were randomly rolled into a control group and a burn group. The control mice were not given any medication and were fed normally. Mice in the burn model were anesthetized by intraperitoneal injection of 50 mg/kg 1% sodium pentobarbital. The back skin was prepared, and the hair was removed; the mice were fixed on the operating table, and the depilated area was scalded continuously for 15 s with 97°C hot water to obtain a third-degree burn model. Immediately after modeling, 1 mL of 0.9% sterile normal saline was intraperitoneally injected for antishock treatment, and the wounds were disinfected with iodophor disinfectant.

#### 2.7.2. Real-Time Fluorescence Quantitative Polymerase Chain Reaction (rt-qPCR)

After 15 days of modeling, the back skin tissue of the same part of the two groups of mice was taken. After the blood was flushed with phosphate buffer, it was snap frozen in liquid nitrogen. After fully grinding the tissue, the Trizol method was used to extract total RNA from the tissue, and the concentration, purity, and integrity of the extracted RNA were detected. Using the extracted RNA as a template, reverse transcription of cDNA was performed according to the instructions of the PrimeScript™ RT reagent Kit with gDNA Eraser (perfect real-time) kit (Takara, Japan). Then, quantitative detection of the target gene was performed according to the instructions of the TB Green® Premix Ex Taq™ II (Tli RNaseH Plus) kit (Takara, Japan). The reaction system was set as follows: 10 *μ*L TB green Premix Ex Taq™ II reagent, 0.8 *μ*L upstream primer, C0.8 *μ*L downstream primer, 0.4 *μ*L ROX Reference Dye, 2 *μ*L cDNA template, and 6 *μ*L ddH_2_O. Quantitative primers were designed and synthesized by Shanghai Sangon Bioengineering Co., Ltd. The primer information was shown in Table 1.

#### 2.7.3. Western Blot

The tissue was crushed thoroughly, and RIPA reagent was applied for protein extraction in the frozen skin tissue from the back of the mouse. The protein concentration of the extracted sample was determined according to the instructions of the BCA kit, the corresponding stacking gel and separating gel were prepared, and the sample protein was loaded and electrophoresed. After the target protein band was transferred to the membrane, a blocking solution containing 5% nonfat milk powder was used for blocking treatment at room temperature for 1 hour. After washed, add diluted primary antibodies; rabbit monoclonal STAT1 (1 : 2000), rabbit monoclonal JUN (1 : 5000), rabbit monoclonal Bcl2 (1 : 2000), rabbit monoclonal MMP9 (1 : 2000), rabbit monoclonal TLR2 (1 : 1000), and mouse monoclonal *β*-actin (1 : 5000) were incubated at 4°C for 12 hours. After recovery of the antibody, it can add the diluted secondary antibody, horseradish peroxidase-labeled goat anti-mouse IgG (1 : 10000), and incubate at room temperature for 1 hour in the dark. In addition, the target protein band was developed according to the instructions of the ECL chemiluminescence kit. The ImageJ software in the gel imager was adopted to measure the gray value of the target protein band, and *β*-actin was undertaken as the internal reference gene to detect the relative expression level of the target protein.

## 3. Statistical Analysis

SPSS 22.0 was used for data processing and statistical analysis. In the rt-qPCR detection results, the 2^−△△CT^ method was applied to calculate the relative mRNA expression level of target gene, where △CT value = CT_target gene_ − CT_internal reference gene_, 2 − △△CT = △CT_burn group_ − △CT_control group_. The relative expression levels of mRNA and protein were compared between groups using independent samples *t* test, and expressed as mean ± standard deviation. *p* < 0.05 was considered to be statistically significant.

## 4. Results

### 4.1. Construction of WGCNA Network

Screening from the dataset, 563 DEGs were obtained, and the volcano plot of DEGs was shown in Figure 3. As it was given, the clustering results of the genes screened from the dataset had no obvious outlier samples, so they can be included in the subsequent WGCAN.

To improve the analysis effect of constructing the WGCNA model, the relationship between the soft threshold and the correlation coefficient (the left of Figure 4) and the relationship between the soft threshold and the mean value of the gene connection coefficient (the right of Figure 4) were plotted. It can be found that when the weighting coefficient *β* (i.e., soft threshold) in the WGCNA model was 9, the correlation coefficient and gene average connection coefficient of the constructed model were optimal. Therefore, *β* = 9 was subsequently set for analysis.

### 4.2. Clinical Correlation Analysis Based on WGCNA Network

The correlation between external information and network modules was found from the gene coexpression network, and then, the network modules with high similarity were found. When *β* = 9 in the WGCNA network, the squared value of the correlation coefficient between log (*k*) and log [*p*(*k*)] was greater than 0.9, and then, the constructed WGCNA network is shown in Figure 5.

Subsequently, the correlation heat map and cluster analysis of the WGCNA network module were constructed, and the results were given in Figure 6. As the figure revealed, 10 corresponding modules were screened in this work, and the clinical characteristics were highly correlated with the green, brown, and gray modules in the WGCNA network.

### 4.3. Analysis on Burn DEGs Based on WGCNA Network

The WGCNA network was utilized to determine the key and differentially expressed genes, and Gene Ontology and KEGG tools were employed to undertake functional annotation of DEGs and enrichment analysis of signaling pathways.  Figure 7 depicts the outcomes. As can be known from Figure 7(a), DEGs were mainly enriched for molecular functions such as replicative senescence, bacterial response to acyl bacterial lip peptides, and Toll-like receptor signaling pathways. They were mainly enriched for biological processes such as CCR5 chemokine receptor binding, histone kinase activity, and lipopeptide binding, and they were enriched for cell components such as cyclin B1-cdk1 complex and dependent protein kinase holoenzyme complex. As demonstrated in Figure 7(b), DEGs were mainly located in the PD-1/PD-L1 pathway, the AGE-RAGE pathway, the Toll-like receptor signaling pathway, the p53 signaling pathway, or the NF-*κ*B signaling pathway.

The genes highly related to burns were found through the identification module, and the top 10 DEGs were selected using functional clustering analysis. The results were illustrated in Table 2. The top 10 DEGs were mainly located in the green, brown, and gray modules of the WGCNA network.

### 4.4. Analysis on Protein Interaction Network of DEGs in Burn Tissue

The protein-protein interaction network of DEGs was constructed using STRING online software, and the results are illustrated in Figure 8.  Figure 8(a) revealed the overall analysis results of DEGs protein-protein interaction network. Except for STEAP4, LMO7, BTBD17, and AMPD3 genes that were not related to other genes, there was an interaction among the proteins of other genes.

JUN, STAT1, Bcl2, MMP9, and TLR gene subprotein were selected for the construction of protein interaction network.  Figure 8(b) suggested that the JUN gene was closely related to CTNNB1, EP300, SMAD3, ATF2, FOS, FOSL1, BATF3, ATF3, and FOSL2. STAT1 gene was closely related to IFNGR1, JAK2, IRF9, IFNAR1, IRF1, JAK1, CREBBP, EP300, PIAS1, and KPNA1. The Bcl2 gene was closely correlated to BBC3, TP53, Bcl2L11, BAX, BAD, BIK, BID, Bcl2L1, FKBP8, and BECN1. MMP9 gene was closely correlated with CD44, TIMP1, SDC1, CDH1, VEGFA, PLG, TIMP3, TGFB1, LCN2, and IL6. TLR2 gene was closely related to IRAK1, HMGB1, LY96, CLEC7A, HSP90B1, HSPD1, VCAN, CD14, TollIP, and TIRAP.

### 4.5. Identification of Burn DEGs

First, rt-qPCR was used to detect the differences in the mRNA expression levels of STAT1, JUN, Bcl2, MMP9, and TLR2 in the burn tissue of mice in the control group and the burn group. The results demonstrated in Figure 9 revealed that compared with the control group, the mRNA expression levels of STAT1 and Bcl2 in the burn group were decreased, while those of JUN, MMP9, and TLR2 were increased (*p* < 0.05).

Western blot detected the differences in PELs of STAT1, JUN, Bcl2, MMP9, and TLR2 in the tissues of mice, and the results were shown in Figure 10. Compared with the control group, the PELs of STAT1 and Bcl2 in the burn group were decreased, while the PELs of JUN, MMP9, and TLR2 were greatly increased (*p* < 0.05).

## 5. Discussion

Burn is a very common disease, and most patients have burns of grade 2 and above [18]. Scar is one of the most common complications of burn patients during rehabilitation, which seriously affects the rehabilitation effect and quality of life of patients [19]. Therefore, this work is of great significance to explore the potential therapeutic targets in the process of wound healing after burn injury and to improve the prognosis of burn patients. In this work, based on WGCNA analysis, the related gene modules of wound healing after burn were searched, and the expression status of DEGs was explored by bioinformatics analysis method, aiming to provide reference materials for the improvement of wound healing effect.

Based on WGCNA, multiple DEGs were obtained, and Gene Ontology functional annotation of these genes [20] and enrichment analysis of KEGG signaling pathway [21] were performed. The results of Gene Ontology analysis showed that DEGs after burn were related to immune system function, metabolic process, and cellular biological regulation. The results of KEGG pathway enrichment analysis showed that DEGs after burn were mainly located in the Toll-like receptor [22], p53 [23], PD-1/PD-L1 [24], and NF-*κ*B [25]. Toll-like receptor signaling pathway can activate bacterial membrane components and promote the activation of MAPK signaling pathway, which in turn triggers the body's inherent immune response and increases the production of proinflammatory factors [26].

Subsequently, five DEGs were screened for expression level verification. The STAT protein family can participate in the binding of different cytokines or growth factors, which can be activated by a variety of cytokines and mediate the expression of multiple genes in response to pathogen invasion [27]. STAT1 plays an important role in antigen presentation and B cell development [28]. Studies have shown that the decrease in the expression level of STAT1 can lead to a decrease in the expression level of IgG, which in turn increases the susceptibility of the body to the virus [29]. JUN is a stress-activated protein kinase, which plays an important role in the process of apoptosis [30]. Studies have confirmed that after inhibiting the expression of JUN, the content of proinflammatory factors such as IL-6 will also decrease, while the content of anti-inflammatory factors such as IL-10 will increase [31]. Bcl2 is also one of the serious hot spots in the process of apoptosis, and it mainly plays the role of inhibiting apoptosis and promoting apoptosis [32]. MMP9 can activate the functions of cytokines and chemokines, so it is involved in the processes of skin wound inflammatory response, matrix remodeling, and epithelialization [33]. Toll-like receptors can selectively recognize microorganisms and their tissue components, and TLR2 plays an important role in the activation of cells by Gram-positive bacteria [34]. The results of this work suggested that the expression levels of STAT1 and Bcl2 in burn tissue were much lower than compared to the normal tissue, while the levels of JUN, MMP9, and TLR2 were remarkably higher. The above results suggest that the body after burn may inhibit the proliferation of immune cells, promote cell apoptosis, reduce the body's immunity, and then, reduce the resistance to external pathogens. The increased expression of JUN in burn tissue triggers the excessive release of proinflammatory factors in the body, which in turn leads to a severe inflammatory response in the body. Therefore, the continuous high expression of inflammatory factors such as JUN, MMP9, and TLR2 in burn wounds tissue may slow down the speed of wound healing.

## 6. Conclusions

WGCNA and other bioinformatics analysis approaches were used to investigate the features of DEGs in burn tissue in this study. According to the WGCNA mining results, ten network modules were discovered to be strongly associated to postburn wound healing, with the green, brown, and grey modules having the most DEGs. The Gene Ontology and KEGG analysis of DEGs found that these genes were mainly functionally annotated as immune cell activation, inflammatory response, and immune response, etc., and were mainly enriched in PD-1/PD-L1, Toll-like receptor signaling, p53, and NF-*κ*B. Later, it was found that the wound healing effect after burn was closely related to genes such as STAT1, JUN, Bcl2, MMP9, and TLR2. However, it only used published data to analyze gene coexpression networks in this work. Clinical tissue samples would be acquired for transcriptase analysis in the follow-up study, and WGCNA would be built and examined again. The results of this work were aimed at finding potential targets for wound healing after burns and providing reference data for improving the prognosis of burn patients.

## Figures and Tables

**Figure 1:** The specific analysis process of WGCNA.

**Figure 2:** The specific flow of burn-related gene analysis using WGCNA.

**Figure 3:** Volcano plot analysis of DEGs. Genes with no statistically great difference were marked in black, genes with low expression and statistically obvious difference were marked in green, and genes with high expression and statistically remarkable difference were marked in red.

**Figure 4:** Soft threshold determination of WGCNA networks.

**Figure 5:** WGCNA network module of DEGs in burn tissue and normal tissue.

**Figure 6:** Modules of WGCNA network and its interaction analysis with clinical characteristics. (a) The interaction among different network modules and (b) the association between network modules and clinical features.

**Figure 7:** Gene Ontology and KEGG analysis of DEGs. (a) The Gene Ontology analysis result of DEGs and (b) the KEGG analysis result of DEGs.

**Figure 8:** DEGs have a complex protein interaction network. The total protein-protein interaction network was depicted in (a); (b) diagram of the subprotein-protein interaction network, where A was the JUN gene, B was the STAT1 gene, C referred to the Bcl2 gene, D represented the MMP9 gene, and E stood for the TLR2 gene.

**Figure 9:** Detection results of mRNA expression levels of DEGs. (a–e) The detected values of STAT1, JUN, Bcl2, MMP9, and TLR2, respectively, and ∗ indicated a statistically obvious difference between groups (*p* < 0.05).

**Figure 10:** Detection results of PELs of DEGs. (a–f) The detected values of STAT1, JUN, Bcl2, MMP9, and TLR2, respectively, and ∗ indicated a statistically obvious difference between groups (*p* < 0.05).

**Table 1:** The quantitative primers of DEGs.

Gene name	Primer sequence (5′→3′)	Size of product (bp)
STAT1 decreased	F: TACGGAAAAGCAAGCGTAATCT	219
	R: TGCACATGACTTGATCCTTCAC	
JUN increased	F: GTGTGGGACGACGATCAAAAG	151
	R: TGACCACTAACAGGGAAGGAC	
Bcl2 decreased	F: ACGTGGACCTCATGGAGTG	129
	R: TGTGTATAGCAATCCCAGGCA	
MMP9 increased	F: GCAGAGGCATACTTGTACCG	229
	R: TGATGTTATGATGGTCCCACTTG	
TLR2 increased	F: CTCTTCAGCAAACGCTGTTCT	237
	R: GGCGTCTCCCTCTATTGTATTG	
GAPDH	F: TGGCCTTCCGTGTTCCTAC	178
	R: GAGTTGCTGTTGAAGTCGCA	

**Table 2:** Information of the top 10 DEGs.

Gene ID	Gene	Full name of the gene	Module	Regulation
ENSG00000177606	JUN	Jun protooncogene	Green	Up
ENSG00000115415	STAT1	Signal transducer and activator of transcription 1	Grey	Down
ENSG00000171791	Bcl2	BCL2 apoptosis regulator	Green	Down
ENSG00000100985	MMP9	Matrix metallopeptidase 9	Green	UP
ENSG00000137462	TLR2	Toll-like receptor 2	Brown	UP
ENSG00000096968	JAK2	Janus kinase 2	Brown	UP
ENSG00000170458	CD14	CD14 molecule	Green	UP
ENSG00000170312	CDK1	Cyclin-dependent kinase 1	Brown	Up
ENSG00000168610	STAT3	Signal transducer and activator of transcription 3	Brown	Up
ENSG00000177455	CD19	CD19 molecule	Green	Down

## Data Availability

The data used to support the findings of this study are available from the corresponding author upon request.
